# Ultrasound-Guided Percutaneous Transhepatic Gallbladder Drainage Improves the Prognosis of Patients with Severe Acute Cholecystitis

**DOI:** 10.1155/2022/5045869

**Published:** 2022-08-29

**Authors:** Xin Jin, Yunshan Jiang, Jiongjiong Tang

**Affiliations:** Department of Ultrasound Medicine, The Central Hospital of Yongzhou, Yongzhou, Hunan 425006, China

## Abstract

The aim of this study was to investigate the clinical efficacy of ultrasound-guided percutaneous transhepatic gallbladder drainage (PTGD) for the treatment of severe acute cholecystitis (AC). The data of 40 patients diagnosed with severe AC at our hospital between August 2020 and June 2021 were retrieved and classified into a PTGD group, open cholecystostomy (OC) group, laparoscopic cholecystectomy (LC) group, and conventional conservative treatment (CT) group. Before treatment and on days 1, 3, 5, and 7 after treatment, their serum levels of alanine aminotransferase (ALT), alkaline phosphatase (ALP), aspartate aminotransferase (AST), total bilirubin (TBIL), triglyceride (TG), high-density lipoprotein (HDL), low-density lipoprotein (LDL), white blood cell count (WBC), IL-2, IL-4, IL-6, IL-8, and cancer antigen 19–9 (CA19-9) were measured. Additionally, clinical manifestations such as body temperature and pain score were monitored before treatment and at 24, 48, and 72 hours after treatment. The recovery time and complications/adverse reactions were statistically analyzed, and the Kaplan–Meier survival curve was plotted. After treatment, compared with the other three groups, the PTGD group had a significant reduction in serum indicators, including WBC and inflammatory factors, recovery time, pain score, and complications, and benefitted from better treatment efficacy and higher survival rate. Thus, ultrasound-guided PTGD was found to be more effective in treating severe AC patients and was associated with improved patient prognoses.

## 1. Introduction

Humans have long suffered from gallstones. According to research statistics, about 10%–15% of Americans have gallstones [1]. However, most patients with gallstones are asymptomatic. Population-based studies showed that 10–18% of patients with asymptomatic gallstones may experience biliary pain, of whom 7% might require surgical intervention and 1–4% could lead to complications such as acute cholecystitis (AC), gallstone pancreatitis, and choledocholithiasis [2]. It has been reported that the incidence of gallbladder disease increases with age, threatening the health of the aging population [3]. Gallstones sometimes migrate out of the gallbladder, block the normal flow of bile, and cause inflammation and infection of the gallbladder. This resulting condition is called cholecystitis and can lead to persistent and intense abdominal pain, fever, nausea, and vomiting [4].

AC accounts for 14–30% of cholecystectomies [5] and is defined as an inflammation of the gallbladder, usually caused by cystic duct obstruction [6]. The most common causes of cystic duct obstruction are gallstones and cholestasis. Other less common causes include masses (primary tumors or gallbladder polyps), parasites, or foreign bodies. Acute calculous cholecystitis is a common disease that requires surgical treatment. It was reported that approximately 120,000 cholecystectomies are performed in the United States annually [7]. If left treated, AC could lead to persistent obstruction of the cystic duct, causing mucus accumulation due to its continued production, and no outlet for drainage. As a result, the gallbladder pressure increases and venous stasis occurs, followed by arterial stasis and ischemic gallbladder necrosis. Necrotic tissue then causes complications such as gallbladder perforation and empyema.

Laparoscopic cholecystectomy (LC) is currently the gold standard for treating AC [8]. However, cholecystectomy is not suitable for many elderly patients with multiple comorbidities. For patients who are not candidates for surgery, less invasive interventions, such as percutaneous transhepatic gallbladder drainage (PTGD), are performed to reduce surgery-related morbidity and mortality [9]. PTGD is a minimally invasive surgery to decompress the gallbladder and is usually used in critically ill patients [10]. In clinical practice, the indications for PTGD include calculous and acalculous cholecystitis, gallbladder perforation, malignant obstruction, percutaneous gallstone removal, and biliary drainage [11]. In addition, PTGD is often used as one of the auxiliary examination methods for cholangiography, gallstone dissolution, and lithotripsy [12]. In the diagnosis of cholecystitis, imaging examinations such as ultrasound, CT, and hepatobiliary scan are essential for surgery to determine the specific circumstances of the gallbladder, as well as to select the appropriate access for gallbladder decompression [13]. Previous clinical studies showed that the overall success rate of PTGD was higher than 95% [14], achieving a clinical improvement in 56%–93% of patients, with only 3%–13% developing complications such as biliary peritonitis, massive hemorrhage, and hemothorax/pneumothorax [14].

However, the effects of PTGD in treating severe AC patients remain controversial. Thus, in this study, we compared PTGD with other surgical methods to determine its clinical efficacy and impact on the survival of severe AC patients to provide evidence for its clinical significance in severe AC.

## 2. Materials and Methods

### 2.1. Study Subjects

In this study, severe AC was defined as a gallbladder inflammation complicated with acute pain and serum markers abnormalities, such as an increase in WBC levels >15 × 10^9^/L, and diagnosed via imaging. The data of patients diagnosed with severe AC in our hospital between August 2016 and June 2019 were retrospectively retrieved, analyzed, and divided into four groups based on their treatment methods, namely, the ultrasound-guided PTGD group (PTGD, *n* = 14), open cholecystostomy group (OC, *n* = 12), LC group (LC, *n* = 8), and conventional conservative treatment group (CT, *n* = 6). The study inclusion criteria were as follows: (1) all patients underwent color Doppler ultrasound, CT, or MRI to confirm the diagnosis; (2) did not receive any treatments, such as antibiotics, prior to diagnosis; and (3) had typical clinical manifestations of AC such as the presence of fever/shivering, right upper abdominal pain/tenderness, diffuse pain/tenderness, nausea/vomiting, and/or positive Murphy's sign; and (4) had almost similar postoperative management, unless they had postoperative complications, which were treated on an individualized basis. The exclusion criteria were as follows: (1) the presence of malignant tumors and dysfunction of vital organs; (2) severe systemic infection; (3) gastrointestinal diseases, such as gastrointestinal perforation and bleeding; (4) a history of abdominal surgery; and (5) poor coagulation, mental illness, severe cognitive impairment, or language problems. The baseline data of the patients, including age, gender, body mass index (BMI), onset symptoms, gallbladder diameter, stage of septic shock, site of infection, duration of abdominal pain, and disease history, were recorded. Since this was a retrospective study, the patients' treatments were based on the treating physician's discretion and after consultation with the patients and/or relatives. The study protocol was approved by the Ethics Committee of The Central Hospital of Yongzhou. All the methods were performed in accordance with the Declaration of Helsinki.

### 2.2. Surgical Methods

In the PTGD group, patients were placed in the supine position. Then, the size and location of the gallbladder and surrounding organs were scanned using an ultrasound machine, based on which an appropriate puncture site and puncture route were selected. After anesthetic infiltration into the peritoneum at the puncture site, the gallbladder was punctured using a disposable pigtail drainage catheter under ultrasound guidance. The puncture needle was made to enter the gallbladder cavity, and the outflow of bile was observed. Then, the guidewire was inserted into the gallbladder, and the chest wall was expanded to insert the drainage tube. The extracted bile or pus was connected to a drainage bag, and the fixed line of the drainage tube was tightened. Last, after the drainage tube was fixed, the body surface was sutured. After treatment, routine anti-infection, semiliquid, low-fat food, and other symptomatic and supportive treatment were given.

In the OC group, patients were placed in the supine position. Then, a paramidline incision of about 10 cm in length was made. The drainage tube was inserted in the gallbladder, and the incision was sutured. After treatment, the patients received symptomatic and supportive treatment such as conventional anti-infection and intravenous nutrition.

In the LC group, patients were treated with four-port LC. During the procedure, the conditions of Calot's triangle and abdominal cavity were observed. After clarifying the relationship between the three ducts, the neck and duct of the gallbladder were disconnected. Lastly, the gallbladder was removed using a combined antegrade and retrograde approach, and an abdominal drainage tube was inserted routinely.

In the CT group, surgical treatment was recommended after admission, but the patients and their families refused. Therefore, during hospitalization, the patients only received conventional anti-infective conservative treatment, and symptomatic treatment was performed according to the condition.

### 2.3. Detection of Biochemical Indicators

Fasting serum was collected from all patients on days 1, 3, 5, and 7 after treatment. After 2-h standing, the supernatant was collected after centrifugation at 3500 rpm for 10 min. Then, an automatic biochemical analyzer (Mindray, China) was employed to measure the expression of alanine aminotransferase (ALT), alkaline phosphatase (ALP), aspartate aminotransferase (AST), total bilirubin (TBIL), triglyceride (TG), high-density lipoprotein (HDL), low-density lipoprotein (LDL), and white blood cell count (WBC) in the serum.

### 2.4. ELISA

Fasting serum was collected from all patients on days 1, 3, 5, and 7 after treatment. After 2-h standing, the supernatant was collected after centrifugation at 3500 rpm for 10 min. Then, the corresponding ELISA kits (MULTISCIENCES (LIANKE), China) were utilized to detect the expression of interleukin (IL)-2, IL-4, IL-6, IL-8, and cancer antigen 19–9 (CA19-9) in serum.

### 2.5. Detection of Clinical Indicators

Before treatment and at 24, 48, and 72 hours after treatment, the following clinical indicators were recorded, including pain score, body temperature, systolic blood pressure, and diastolic blood pressure. Additionally, the duration of abdominal pain, recovery time of WBC, operation duration, extubation time, and length of hospital stay were observed after treatment. The occurrence of complications/adverse reactions was also recorded.

### 2.6. Follow-Up

All patients were followed up for 2 years, and the data on patients' survival status were obtained to calculate the survival rate of each treatment group.

### 2.7. Statistical Analysis

All data were statistically analyzed using the SPSS 26.0 software (SPSS Inc., Chicago, IL, USA). Measurement data were expressed as mean ± standard deviation (SD), and one-way analysis of variance (ANOVA) was used for comparison between groups. Enumeration data were expressed as frequency (*n*) and rate (%), and the chi-squared test or Fisher's exact test was used for statistical analysis. Survival curve was plotted using the Kaplan–Meier and compared with the log-rank test. *P* < 0.05 was set as a cutoff for statistical significance.

## 3. Results

### 3.1. Baseline Data of Patients

A total of 40 patients were found eligible for this study. The patients in all groups were over 60 years of age. There were no significant differences in age, gender, BMI, clinical symptoms, time from onset to admission, trigger, history of diseases disease, ASA grade, and APACHE II score among the groups (Table 1). Therefore, the comparability of the patients was ensured.

### 3.2. Comparison of Preoperative Clinical Indicators among the Four Groups

The preoperative clinical parameters were compared, including WBC, neutrophil count, ALT, ALP, AST, TBIL, TG, HDL, LDL, and systolic and diastolic blood pressure. The results showed no significant difference in these indicators among the four groups (Table 2).

### 3.3. Comparison of Postoperative Clinical Indicators among the Four Groups

Their postoperative clinical symptoms were compared, and the results including that the duration of abdominal pain (18.03 ± 3.02), recovery time of WBC (3.21 ± 0.40), operation duration (58.31 ± 10.09), extubation time (2.10 ± 0.40), and length of hospital stay (2.99 ± 1.31) were the shortest in the PTGD group, while the CT group had the worst effect (Table 3).

### 3.4. Comparison of Postoperative Serum Indicators at Different Time Points among the Four Groups

Clinical biochemical parameters and inflammatory factors were measured on days 1, 3, 5, and 7 after treatment in the four groups. The results showed that the ALT, AST, ALP, TBIL, WBC, and CA19-9 on days 3, 5, and 7 after treatment in the four groups gradually decreased compared with Day 1 and returned to the normal range, with the PTGD group demonstrating the most significant decrease (Figure 1(a)). Further examination of the serum levels of inflammatory factors in the four groups showed that the IL-2, IL-6, and IL-8 and IL-4 levels in the four groups also gradually returned to the normal range on 3, 5, and 7 days after treatment compared with Day 1. Compared with the other groups, the PTGD group had the lowest expression of inflammatory factors and the highest expression of anti-inflammatory factors from day 1 to day 7 after treatment (Figure 1(b)).

### 3.5. Comparison of Postoperative Complications among the Four Groups

The results showed that all four groups had some complications or adverse reactions after treatment. The patients in the PTGD group mainly had four complications, including wound infection (*n* = 1), stress ulcer (*n* = 1), urinary tract infection (*n* = 2), and incomplete intestinal obstruction (*n* = 1). Seven kinds of complications or adverse reactions occurred in the other three groups, with the CT group having the highest number of complications than the other groups. For instance, the results showed that the probability of upper gastrointestinal bleeding in the CT group was as high as 50%. Overall, the PTGD group had the lowest probability of complications (Table 4).

### 3.6. Comparison of Survival among the Four Groups

Forty patients were followed up for two years, and their survival status and duration were analyzed. The results showed that during follow-up, there were 2 deaths (14.3%) in the PTGD group, 4 deaths (33.3%) in the LC group, 4 deaths (50%) in the OC group, and 4 deaths (66.7%) in the CT group (Figure 2). Thus, the survival rate of the PTGD group was the highest (85.7%), while the CT group showed the lowest survival rate (33.3%).

### 3.7. Typical Case Report of Severe AC from Hospitalization to Discharge

A 38-year-old woman was hospitalized in our hospital for 3 days with persistent distending pain in the upper abdomen, no pain radiating to other parts of the body, no correlation between pain and position change, no self-remission after rest, and absence of nausea, vomiting, diarrhea, chills, fever, and acid reflux. Physical examination showed that the pressure pain was located in the epigastrium and subxiphoid process, with percussion pain in the liver area. No rebound tenderness or obvious mass was observed, and the liver and spleen were not enlarged. An abdominal ultrasound showed that the diameter of the gallbladder was 200 × 48 mm (Figure 3). Based on these observations, acute severe cholecystitis was considered, and the patient underwent ultrasound-guided percutaneous transcatheter gallbladder puncture placement. She was placed in a supine position. After routine disinfection, real-time color ultrasound was used to guide and monitor the needle entry to avoid large vessels. It passed through a portion of liver tissue, and after its tip reached the gallbladder, the needle core was withdrawn, and brown viscous bile was aspirated. Then, the support was removed, and the traction line was pulled. After successfully placing the catheter, it was externally fixed (Figure 4). Following this procedure, the patient's abdominal distention and discomfort were significantly relieved, and she was discharged on the third day of hospitalization.

## 4. Discussion

Our results showed the levels of ALT, AST, ALP, TBIL, WBC, and CA19-9 in all four treatment groups gradually decreased from Day 1 to Day 7, with the PTGD group demonstrating the most significant decrease, and the levels of IL-2, IL-6, IL-8, and IL-4 gradually returned within normal ranges, with the PTGD group demonstrating the lowest expression of inflammatory factors and highest expression of anti-inflammatory factors. These findings indicate that ultrasound-guided PTGD was the most effective treatment for AC patients, at least in this present study. AC is an acute inflammation triggered by cystic duct obstruction caused by various factors [15]. Studies have shown that ultrasound-guided PTGD has a high success rate in elderly AC patients and was associated with a low level of inflammation after surgery [16], which was concordant with the results of our study.

Like most inflammatory diseases, AC is usually associated with leukocytosis, but the manifestations may vary in different patients [17]. According to statistics, 32–53% of patients have fever when they come to the hospital, and 51–53% have leukocytosis [6]. In this study, we found that after treatment, the level of WBC was decreased in all four groups compared with before treatment, and the decrease was most prominent in the PTGD group, while it was least favorable in the CT group. Kim et al. also reported that PTGD could rapidly reverse local inflammation and reduce its systemic effects in patients who could not undergo surgery due to severe comorbidities [18].

Recently, ultrasound-guided PTGD has received significant attention as a potential method of internal gallbladder drainage and is indicated for high-risk patients who cannot undergo cholecystectomy [19]. This study confirmed that ultrasound-guided PTGD was associated with the shortest operation duration, extubation time, and length of hospital stay compared with the other three treatments. This could be because ultrasound-guided PTGD can be effectively performed with ultrasound assistance to directly observe the whole procedure, thereby reducing the risk of complications. Therefore, compared with traditional conventional surgery, ultrasound-guided PTGD is associated with more accurate localization, a clearer field of vision, less trauma, and lower risk of complications [20]. In our typical case, a middle-aged woman was hospitalized due to persistent epigastric pain and discomfort. After completing relevant examinations, she was diagnosed with acute severe cholecystitis and was immediately treated with ultrasound-guided percutaneous transcatheter cholecystocentesis, during which the patient's vital signs were stable. In a randomized study of 61 patients, it was observed that patients treated with PTGD had a shorter hospital stay than those who received LC after conservative treatment [21]. Regarding the treatment response rate, this study also found that patients in the PTGD group had the best prognosis among the four groups. Another randomized controlled trial, including 58 severe AC patients, demonstrated that PTGD was clinically effective in 90% of patients, while OC was effective in 61% of patients [22]. In addition, a systematic review of PTGD for AC patients reported that PTGD was clinically successful, with 85.6% of the patients showing clinical improvement within 48–72 hours, and only 6.24% experienced adverse events. Although the mortality related to the surgery was only 0.36%, the overall mortality was 15% [23]. In contrast to our study, patients in the PTGD group had the lowest incidence of complications and adverse reactions.

The efficacy and safety of PTGD are still somewhat controversial. A study reported that in a case series of high-risk elderly AC patients, the mortality rate of cholecystectomy was 0%, while that of PTGD was 17.2% [24]. The main reason for such controversy could be that the guiding modalities for PTGD were different. PTGD, according to multiple meta-analyses, is reliable under ultrasound guidance, and even ultrasound-guided PTGD has higher success rates and lower readmission and reintervention rates, with a 1-year adverse event rate relative to other modalities [25–28].

Despite the clinically important results in this study, some limitations have to be mentioned. First, this study was limited due to its retrospective nature and small cohort size. Second, the follow-up time was relatively short, and long-term follow-ups are required to further confirm the efficacy of PTGD. Third, this was a single-center study based on Chinese patients, and whether these observations would be similar in a multicenter and multiethnicity cohort remained to be determined.

## 5. Conclusion

In summary, compared with open cholecystostomy, LC, and conventional conservative treatment, ultrasound-guided PTGD was associated with the greatest normalization of serum indicators, fastest recovery time, lowest risk of complications, and highest survival rate; supporting the clinical application of PTGD in severe AC patients. However, due to the limited number of cases and additional limitations, further investigations in multicenter prospective settings are required to confirm the efficacy of PTGD.

## Figures and Tables

**Figure 1:** Comparison of serum indicators at different time points after treatment among the four treatment groups. (a) Serum ALT, AST, ALP, TBIL, WBC, and CA19-9 levels on days 1, 3, 5, and 7 after treatment. (b) Serum IL-2, IL-4, IL-6, and IL-8 levels on days 1, 3, 5, and 7 after treatment. ^*∗*^*P* < 0.05, ^*∗∗*^*P* < 0.01*vs*. the CT group, ^##^*P* < 0.01*vs*. the LC group. PTGD, percutaneous transhepatic gallbladder drainage; LC, laparoscopic cholecystectomy; OC, open cholecystostomy; CT, conventional conservative treatment.

**Figure 2:** Comparison of survival among the four treatment groups.

**Figure 3:** Illustration of an enlarged gallbladder, of size approximately 200 × 48 mm.

**Figure 4:** Illustration of a successfully cannulated gallbladder. The catheter was successfully punctured into the gallbladder, as indicated by the red arrow.

**Table 1:** Baseline data of the severe acute cholecystitis patients included in this study.

Variables	PTGD (*n* = 14)	LC (*n* = 12)	OC (*n* = 8)	CT (*n* = 6)	*P* value
Age (year)	62.5 ± 12.0	63.3 ± 13.9	66.5 ± 9.9	60.8 ± 15.7	NS
Gender (male/female)	6/8	7/5	3/5	3/3	NS
BMI (kg/m^2^)	28.23 ± 5.02	26.78 ± 6.03	28.23 ± 6.93	26.03 ± 4.02	NS

Clinical symptoms/signs (*n* (%))					
Fever/shivering	10 (71.4)	8 (66.7)	5 (62.5)	4 (66.7)	NS
Right upper abdominal pain/tenderness	13 (92.9)	12 (100.0)	7 (87.5)	6 (100.0)	NS
Diffuse pain/tenderness	7 (50.0)	5 (41.7)	5 (62.5)	2 (33.3)	NS
Nausea/vomiting	5 (35.7)	4 (33.3)	3 (37.5)	3 (50.0)	NS
Positive Murphy's sign	8 (57.1)	5 (41.7)	3 (37.5)	3 (50.0)	NS
Time from onset to admission (d)	4.0 ± 1.5	3.5 ± 1.3	4.5 ± 1.7	4.3 ± 2.5	NS

Trigger (*n* (%))					
Calculous	10 (71.4)	8 (66.7)	7 (87.5)	4 (66.7)	NS
Noncalculous	4 (28.6)	4 (33.3)	1 (12.5)	2 (33.3)	NS
Thickness of gallbladder wall (cm)	0.68 ± 0.23	0.73 ± 0.26	0.66 ± 0.30	0.70 ± 0.34	NS

History of diseases (*n* (%))					
Cardiovascular diseases	9 (64.3)	6 (50.0)	5 (62.5)	4 (66.7)	NS
Lung diseases	3 (21.4)	2 (16.7)	2 (25.0)	1 (16.7)	NS
Diabetes	4 (28.6)	2 (16.7)	3 (37.5)	2 (33.3)	NS
Chronic kidney disease	2 (14.3)	1 (8.3)	1 (12.5)	1 (16.7)	NS

ASA grade (*n* (%))					
≤II	5 (35.7)	4 (33.3)	4 (50.0)	2 (33.3)	NS
III-IV	9 (64.3)	8 (66.7)	4 (50.0)	4 (66.7)	NS
APACHE II score (point)	15.6 ± 3.6	14.2 ± 4.5	13.6 ± 2.8	14.7 ± 3.5	NS

Note: PTGD, percutaneous transhepatic gallbladder drainage; LC, laparoscopic cholecystectomy; OC: open cholecystostomy; CT, conventional conservative treatment; BMI, body mass index.

**Table 2:** Comparison of preoperative clinical indicators among the four treatment groups.

Variables	PTGD (*n* = 14)	LC (*n* = 12)	OC (*n* = 8)	CT (*n* = 6)	*P* value
WBC (×10^9^/L)	16.71 ± 3.60	15.89 ± 2.49	16.30 ± 3.98	17.10 ± 4.56	0.898
Neutrophil count (%)	88.68 ± 6.64	88.05 ± 7.15	89.76 ± 5.32	88.82 ± 6.50	0.954
ALT (U/L)	73.35 ± 30.04	70.10 ± 29.03	76.35 ± 24.99	72.49 ± 32.05	0.973
ALP (U/L)	142.96 ± 32.76	140.66 ± 36.12	139.64 ± 30.09	138.17 ± 31.30	0.991
AST (U/L)	81.22 ± 24.92	77.81 ± 22.06	79.35 ± 26.20	83.52 ± 31.11	0.970
TBIL (*μ*mol/L)	41.67 ± 11.7	38.35 ± 12.89	38.91 ± 14.2	44.57 ± 16.14	0.767
TG (mmol/mL)	3.21 ± 0.40	3.29 ± 0.45	3.27 ± 0.36	2.9 ± 0.25	0.184
HDL (mmol/mL)	0.9 ± 0.25	0.91 ± 0.30	0.89 ± 0.28	0.93 ± 0.23	0.996
LDL (mmol/mL)	3.1 ± 0.7	3.0 ± 0.6	3.2 ± 0.5	2.9 ± 0.6	0.847
Systolic blood pressure (mmHg)	146.64 ± 26.05	145.75 ± 31.97	144.50 ± 28.65	145.93 ± 27.85	0.999
Diastolic blood pressure (mmHg)	93.36 ± 13.11	90.92 ± 11.07	92.38 ± 14.02	94.0 ± 15.10	0.956

Note: PTGD, percutaneous transhepatic gallbladder drainage; LC, laparoscopic cholecystectomy; OC: open cholecystostomy; CT, conventional conservative treatment; WBC, white blood cell count; ALT, alanine aminotransferase; ALP, alkaline phosphatase; AST, aspartate aminotransferase; TBIL, total bilirubin; TG, triglyceride; HDL, high-density lipoprotein; LDL, low-density lipoprotein.

**Table 3:** Comparison of postoperative clinical indicators among the four groups.

Variables	PTGD (*n* = 14)	LC (*n* = 12)	OC (*n* = 8)	CT (*n* = 6)	*P* value
Duration of abdominal pain (h)	18.03 ± 3.02	22.48 ± 3.32	28.46 ± 3.96	31.70 ± 5.94	<0.001^*∗∗∗*^
Recovery time of WBC (d)	3.21 ± 0.40	4.00 ± 1.00	5.54 ± 2.01	7.00 ± 2.20	<0.001^*∗∗∗*^
Operation duration (h)	58.31 ± 10.09	66.07 ± 12.12	71.65 ± 14	83.58 ± 23.12	0.005^*∗∗*^
Extubation time (h)	2.10 ± 0.40	2.59 ± 0.59	2.98 ± 1.01	4.18 ± 1.49	<0.001^*∗∗∗*^
Length of hospital stay (d)	2.99 ± 1.31	3.99 ± 1.1.51	5.99 ± 2	8.07 ± 2.98	<0.001^*∗∗∗*^

Note: ^*∗∗∗*^*P* < 0.001 vs. CT group; PTGD, percutaneous transhepatic gallbladder drainage; LC, laparoscopic cholecystectomy; OC: open cholecystostomy; CT, conventional conservative treatment; WBC, white blood cell count.

**Table 4:** Comparison of postoperative complications among the four treatment groups.

Complication (*n* (%))	PTGD (*n* = 14)	LC (*n* = 12)	OC (*n* = 8)	CT (*n* = 6)	*P* value
Wound infection	1 (7.14)	2 (16.7)	3 (37.5)	0 (0.0)	0.198
Upper gastrointestinal bleeding	0 (0.0)	1 (8.3)	2 (25.0)	3 (50.0)	0.026
Stress ulcer	1 (7.14)	4 (33.3)	3 (37.5)	4 (66.7)	0.045
Urinary tract infection	2 (14.3)	0 (0.0)	0 (0.0)	1 (16.7)	0.350
Incomplete intestinal obstruction	1 (7.14)	1 (8.3)	2 (25.0)	2 (33.3)	0.346
Infectious pneumonia	0 (0.0)	2 (16.7)	1 (12.5)	2 (33.3)	0.206
Acute renal failure	0 (0.0)	1 (8.3)	2 (25.0)	1 (16.7)	0.317
Death during hospitalization	0 (0.0)	1 (8.3)	2 (25.0)	1 (16.7)	0.317

Note: PTGD, percutaneous transhepatic gallbladder drainage; LC, laparoscopic cholecystectomy; OC: open cholecystostomy; CT, conventional conservative treatment.

## Data Availability

The datasets generated and/or analyzed in the experiment are available from the corresponding author upon request.
